This article has been retracted.

# Using a new HSPC senescence model in vitro to explore the mechanism of cellular memory in aging HSPCs

**DOI:** 10.1186/s13287-021-02455-x

**Published:** 2021-08-09

**Authors:** Yongpin Dong, Chunni Guo, Wuxiong Zhou, Wenfang Li, Lina Zhang

**Affiliations:** 1 Institute of Basic Medicine, Shanghai University of Traditional Chinese Medicine, 1200 CaiLun Ave., Pudong, Shanghai, 201203 China; 2 Department of Emergency and Critical Care Medicine, Shanghai Changzheng Hospital, The Second Military Medical University, Shanghai, China; 3 Department of Neurology, Shanghai General Hospital, Shanghai Jiao Tong University School of Medicine, Shanghai, China

**Keywords:** Senescence model, HSPC, Cellular memory, TOPOIIα, UHRF1

## Abstract

**Background:**

Age-associated changes attenuate human blood system functionality through the aging of hematopoietic stem and progenitor cells (HSPCs), manifested in human populations an increase in myeloproliferative disease and even leukemia; therefore, study on HSPC senescence bears great significance to treat hematopoietic-associated disease. Furthermore, the mechanism of HSPC aging is lacking, especially the cellular memory mechanism. Here, we not only reported a new HSPC senescence model in vitro, but also propose and verify the cellular memory mechanism of HSPC aging of the Polycomb/Trithorax system.

**Methods:**

HSPCs (Lin^−^c-kit^+^ cells) were isolated and purified by magnetic cell sorting (MACS). The proportions and cell cycle distribution of cells were determined by flow cytometry; senescence-related β-galactosidase assay, transmission electron microscope (TEM), and colony-forming unit (CFU)-mix assay were detected for identification of the old HSPC model. Proteomic tests and RNA-seq were applied to analyze differential pathways and genes in the model cells. qPCR, Western blot (WB), and chromatin immunoprecipitation PCR (CHIP-PCR) were used to detect the gene expression of cell memory-related proteins. Knockdown of cell memory-related key genes was performed with shRNA interference.

**Results:**

In the model old HSPCs, β-gal activity, cell cycle, colony-forming ability, aging-related cell morphology, and metabolic pathway were significantly changed compared to the young HSPCs. Furthermore, we found the model HSPCs have more obvious aging manifestations than those of natural mice, and IL3 is the major factor contributing to HSPC aging in the model. We also observed dramatic changes in the expression level of PRC/TrxG complexes. After further exploring the downstream molecules of PRC/TrxG complexes, we found that Uhrf1 and TopII played critical roles in HSPC aging based on the HSPC senescence model.

**Conclusions:**

These findings proposed a new HSPC senescence model in vitro which we forecasted could be used to preliminary screen the drugs of the HSPC aging-related hemopathy and suggested cellular memory mechanism of HSPC aging.

**Supplementary Information:**

The online version contains supplementary material available at 10.1186/s13287-021-02455-x.

## Introduction

The mammalian blood system is a highly differentiated and dynamic; most blood cells are the most short-lived and quickly replaced within few days. It is established that most mature blood cells are constantly generated and replaced from hematopoietic stem cells (HSCs) through a series of lineage-committed hematopoietic progenitor cells (HPCs) [1], so mammals maintain hematopoiesis by the activity of thousands of hematopoietic stem and progenitor cells (HSPCs) [1–4]. Although the blood is the definitive self-renewing tissue of the body, it does not escape the aging process. The previous study indicated age-related alterations in the human blood system depend on hematopoietic stem and progenitor cells (HSPCs) aging [5–7]. Hematopoietic aging is manifested in human populations in the form of an increase in myeloproliferative disease, including leukemias, declining adaptive immunity, and greater propensity to anemia. Therefore, a study on hematopoietic stem and progenitor cells (HSPCs) senescence bears great significance to treat hematopoietic associated disease. Furthermore, stem cells are exposed to both intrinsic and extrinsic assault over their lifetime; thus, it has been hypothesized that aging or functional failure of stem cells may limit tissue repair and renewal, thereby contributing to overall organismal aging and life span reduction [8]. Therefore, besides great significance to treat hematopoietic disease, a study on HSC/HSPC senescence also bears great significance to further elucidate the mechanisms of aging.

Aging hematopoietic stem and progenitor cell model in vitro is an important platform to study HSC/HPC senescence and associated diseases [9]. To date, there were some ways to build aging HSC/HSPC models in vitro including old animal models [10], busulfan-induced cell aging model [11], radiation-induced cell aging model [12], and tert-butyl hydroperoxide (t-BHP)-induced cell aging model [13]. However, these ways were limited either by long experimental periods or complicated operation steps. Our study proposed a quick and easy method of obtaining aging HSPC in vitro.

Compared with the other aging theories, the mechanism of HSC/HSPC aging remains less known. Besides the known players such as DNA damage, telomere shortening, and oxidative stress, cellular memory maybe very important in HSC aging process [14, 15]. During the development of multicellular organisms, cells become different from one another by a distinct use of their genetic program in response to transient stimuli, an example being lineage specification in hematopoiesis [16]. Long after such a stimulus has disappeared, cellular memory mechanisms still enable cells to “remember” their chosen fate over many cell divisions. Cellular memory is a dynamic balance between the Polycomb group (PcG) and Trithorax group (TrxG) proteins, then their target genes [14, 17–19]. PcG and TrxG group proteins are essential epigenetic regulators that can maintain stable epigenetic memory of silent states (via PcG) and active states (via TrxG) of their target genes. However, the mechanism of cellular memory including PcG/TrxG system alteration that occurs in the HSPC aging process remains less known. Our previous study demonstrated that the gene expression of PcG and TrxG proteins was significantly altered in HSPCs (Lin^-^c-kit^+^) of old mice [18]. In the present study, based on our new HSPC aging model, we further explored the PcG/TrxG proteins expression alteration and the histone methylation regulatory on their target genes TOPOIIα and UHRF1.

## Materials and methods

### Animals and major regents

Equal numbers of male and female C57BL/6J SPF mice were obtained from Shanghai Sippr-BK Experimental Animal Center [Certificate No. SCXK (Shanghai) 2013-0016]. Young mice were 4 weeks of age and 16–18 g in weight, and old mice were 18 months of age and 25–30 g in weight.

### Reagents

Red blood cell lysis buffer, SA-β-Gal staining kit, and cell cycle detection kit were purchased from Beyotime Biotechnology Co.; Lineage (Lin) Cell Depletion kit and Anti-c-kit (CD117) MicroBead kit were purchased from Miltenyi Biotec Co.; TUNEL Apoptosis Detection Kit (Alexa Fluor 647) was purchased from Shanghai Yeasen Biotechnology Co.; RNA Extraction and Purification kit, Reverse Transcription, and Fluorescence Quantitative PCR kit were purchased from Takara Co. Stemspan Stem Cell Media and Mouse Colony-Forming Unit (CFU) Assays Using MethoCult™ were purchased from Stem cell Co.; mouse SCF, mouse IL-3, and mouse IL-6 were purchased from Novus Biologicals Co.; anti-CD117-PE (3C11) was purchased from Miltenyi Biotec Co.; anti-H3K4me3 (C42D8), anti-H3K27me3 (C36B11), anti-Mll1 (C36B11), anti-Trx (C63C6), anti-Ezh2 (D2C9), and anti-Bmi1 (D42B3) were purchased from CST Co.; anti-Mel18 was purchased from Abcam Co.; lipofectamine 3000 was purchased from Invitrogen Co.; and Opti-MEM was purchased from GIBCO Co.

### Isolation and purification of HSPCs

Mice were sacrificed by cervical dislocation. The femur was elevated, and the bone marrow was rinsed. The filtrate was centrifuged, and the pellet was suspended in red blood cell lysis buffer, centrifuged at 3000 rpm, 5 min. The precipitate was bone marrow mononuclear cells (MNCs) (Fig. 1a). MNCs were suspended in PBS containing EDTA and 0.5% BSA. Then, we got HSPC by using Lin^−^c-kit^+^ immunomagnetic beads sorting technique with lineage cell depletion kits and anti-c-Kit microbeads (Fig. 1b). CD117, also known as c-kit, stem cell factor receptor. It is expressed on the majority of hematopoietic progenitor cells, including multipotent hematopoietic stem cells, committed myeloid precursor cells, erythroid precursor cells, and lymphoid precursor cells. CD117 is also expressed on a few mature hematopoietic cells such as mast cells. So, CD117 MicroBeads (Miltenyi Biotec, Order no: 130-091-224) are developed for the isolation of hematopoietic stem/progenitor cells and a few mature hematopoietic cells. The Lineage Cell Depletion Kit (Miltenyi Biotec, Order no: 130-090-858) is a magnetic labeling system for the depletion of mature hematopoietic cells, such as T cells, B cells, monocytes/macrophages, granulocytes, and erythrocytes and their committed precursors from bone marrow. So, after centrifugation and sorting of Lin-c-Kit+, the Lin-c-Kit+ cells of BMCs are considered to be hematopoietic stem cells/progenitor cells (HSPCs).

**Fig. 1:** HSPCs were effectively isolated and purified by MACS. **a** Schematic illustrates the isolation of mouse bone marrow mononuclear cells (MNCs). **b** For lineage depletion, cells were magnetically labeled with a cocktail of biotinylated antibodies that are against a panel of so-called lineage antigens (CD5, CD45R (B220), CD11b, anti-Gr-1, and Ter-119 antibodies) and anti-Biotin MicroBeads. This labeling procedure leaves the lineage-negative cells undisturbed, thus allowing further separation of lineage^−^ cells. Then, the lineage^−^ cells (lin^−^ cells) were purified by c-Kit MACS, namely lin^-^c-Kit^+^ cells. **c** HSPCs were cultured with a specific modeling medium (stem cell culture medium + 10 ng/mL IL3 + 10 ng/mL IL6 + 30 ng/mL SCF) and incubated for 8 days, its the model group. **d** Flow cytometric analysis of the purity of lin–c-Kit+ cells at different phases. The results were expressed as mean ± S.D., and the p values (*P < 0.05, **P < 0.01, ***P < 0.001) were determined by the ANOVA test

All the animal experiments were performed in compliance with the guidelines of the Animal Care and Use Committee of Shanghai University of Traditional Chinese Medicine.

### Flow cytometry analysis

Cellular purity was detected with flow cytometer before and after sorting: to test HSPCs purity, 10^6^ MNCs (unpurified) and 10^6^ Lin^−^c-kit^+^ MNCs (purified) were collected. Ten microliters of CD117-PE was added to the cells. The cells were resuspended in FACS buffer and analyzed by flow cytometry using a Becton Dickinson Accuri™ C6.

### The establishment and identification of old HSPC model

1. Young group: HSPCs were isolated from 4-week-old mice according to the steps above.
2. In vitro senescence model group: Young HSPCs were cultured with the modeling medium [Stemspan Stem Cell Media + 10 ng/mL interleukin 3 (IL3) + 10 ng/mL interleukin 6 (IL6) + 30 ng/mL stem cell factor (SCF)] for 8 days (Fig. 1c). The modeling medium was changed every 2 to 3 days.
3. Old mouse group: HSPCs were isolated from 18-month-old mice according to the steps above.

### SA-β-gal staining

HSPCs (~ 1,000,000 cells) were collected on days 2, 4, 6, and 8. They were all fixed with 4% paraformaldehyde for 15 min. The cells were incubated at 37 °C without CO_2_ for 16 h in a β-galactosidase staining solution. The number of β-galactosidase-positive cells per 400 total cells was counted.

### Cell cycle

HSPCs (~ 1,000,000 cells) were collected, fixed with cold 4% paraformaldehyde for 1 h, and fixed with 70% ethanol overnight at 4 °C. Cells were then incubated in a propidium iodide staining solution (Beyotime) for 30 min at 37 °C in the dark. The cell cycle distribution was analyzed by flow cytometry with the FACS Express software.

### Mixed colony-forming unit (CFU-Mix) of HSPC culture

Cells (1.5 × 10^4^) were collected and subjected to CFU culture: Cells were diluted, in duplicate, with IMDM+ 2% FBS and MethoCult™ GF M3434 medium to a final concentration of 5 × 10^3^ per 35 mm dish. 0.3 mL of the diluted cells were added to 3 mL of MethoCult™ and mixed thoroughly. The final cell mixture was dispensed into each 35 mm dish at a volume of 1.1 mL and incubated at 37 °C in 5% CO_2_ for 7 days. Photos were taken using an inverted microscope. Finally, we added 1 mg/mL p-iodonitrotetrazolium violet to 24-well cells so as to take photos 24 h later. The number of CFU-Mix per 5 × 10^3^ cells represented the pluripotency of the HSPCs.

### Transmission electron microscope (TEM)

Cells (~ 1,000,000 cells) were prefixed with 2.5% glutaraldehyde and then dehydrated with an ethanol gradient series before being embedded in Epon812. Samples were cut into 50–70-nm-thick sections by a microtome. All samples were observed under a transmission electron microscope (TEM) (JEM- 2100, JEOL, Japan).

### Isobaric tags for relative and absolute quantification (iTRAQ)

Protein digestion and iTRAQ labeling were performed as described previously [20]. Briefly, 100 μg of protein from each sample was reduced, alkylated, and then digested with sequence-grade modified trypsin (Promega, Madison, WI) prior to labeling with one of the individual 8-plex-iTRAQ tags (Applied Biosystems, Framingham, MA). The peptide mixture was fractionated by high pH separation using Ultimate 3000 system (Thermo Fisher Scientific, MA, USA) connected to a reverse-phase column (XBridge C18 column, 4.6 mm × 250 mm, 5 μm, Waters Corporation, MA, USA). Twelve fractions were separated by nanoLC and analyzed by online electrospray tandem mass spectrometry. The experiments were performed on an Easy-nLC 1000 system (Thermo Fisher Scientific, MA, USA) connected to a Q-Exactive mass spectrometer (Thermo Fisher Scientific, MA, USA) equipped with an online nano-electrospray ion source. PEAKS DB was set up to search the UniProt mouse database (ver.201711, 51946 entries) assuming the digestion enzyme trypsin. Differently expressed proteins were filtered if their fold changes were over 1.5 and contained at least 2 unique peptides with P (PEAKSQ) below 0.01.

### RNA-seq, library generation, and bioinformatics analysis

HSPCs (~ 1,000,000 cells) were collected. Total RNA was isolated using the RNeasy mini kit (Qiagen, Germany). Strand-specific libraries were prepared using the TruSeq® Stranded Total RNA Sample Preparation kit (Illumina, USA). Briefly, mRNA was enriched with oligo (dT) beads. Following purification, the mRNA is fragmented into small pieces using divalent cations under 94 °C for 8 min. The cleaved RNA fragments are copied into first-strand cDNA using reverse transcriptase and random primers. This is followed by second-strand cDNA synthesis using DNA PolymeraseI and RNaseH. These cDNA fragments then go through an end repair process, the addition of a single “A” base, and then ligation of the adapters. The products are then purified and enriched with PCR to create the final cDNA library. Purified libraries were quantified by Qubit® 2.0 Fluorometer (Life Technologies, USA) and validated by Agilent 2100 bioanalyzer (Agilent Technologies, USA) to confirm the insert size and calculate the mole concentration. Cluster was generated by cBot with the library diluted to 10 pM and then were sequenced on the Illumina HiSeq X ten (Illumina, USA). The library construction and sequencing were performed at Shanghai Biotechnology Corporation, Shanghai, China. For GO enrichment analysis, selected differentially regulated genes between young group and old group HSPCs with a Fisher test-corrected P < 0.05 were analyzed on the Gene Ontology Consortium website (geneontology.org). Like GO enrichment, the association of the genes with different pathways was computed with the Kyoto Encyclopedia of Genes and Genomes (KEGG) (http://www.genome.jp/kegg) databases. All data are representative of three independent experiments.

### TrxG/PcG disequilibrium

#### Quantitative RT-PCR

Quantitative real-time polymerase chain reaction (qRT-PCR) was used to verify the gene expression of PCG proteins (Ezh2, Bmi-1, Eed, MEL18, Rae-28) and TRXG proteins (Mll, Trx). Total RNA extraction and reverse transcription were performed according to the manufacturer’s instructions of the kits (9108/9109, Takara; RR047A, Takara). The A260/280 ratio of RNA was detected. The primers were designed and synthesized by Sango Biotech. The β-actin (internal control) primers were used. All primer sequences are listed: β-actin (internal control): 5′-AACGCAGCTCAGTAACA GT CC-3′ (forward), β-actin (internal control): 5′-GTACCACCATGTACCCAGGC-3′ (reverse); Ezh2: 5′-AGCAGTAAGAGCAGCAGCAA-3′ (forward), Ezh2: 5′-TTCCTTCCATGC AA CACCCA-3′ (reverse); Bmi-1: 5′-GGACTGGGCAAACAGGAAGA-3′ (forward) Bmi-1: 5′-GACTCTGGGAGTGACAAGGC-3′ (reverse); Eed: 5′-GCTCAGCCTGATCGAATG CT-3′ (forward), Eed: 5′-TTGGCGATGGGATCGACTTC-3′ (reverse); Mel18: 5′-TCCCC ATCTCCATTCTCCGT-3′ (forward), Mel18: 5′-ATACCCCCTGACAGAGGTCC-3′ (reverse); Rae-28: 5′-GCACAGATCTTGAGAGCAGG-3′ (forward), Rae-28: 5′-GCAA GGCTGCCAAGAGATTG-3′ (reverse); Trx: 5′-TAAAGCAGTGGCTTAGGGGAC-3′ (forward), Trx: 5′-GAGAGTCTATACCCAACTGCCA-3′ (reverse); and Mll: 5′-ACGCT TG TCTGTCTGGATGG-3′ (forward), Mll: 5′-CCCATGAGATTCCGGCACTT-3′ (reverse).

SYBR green dye was used for real-time quantitative PCR (RR420A, Takara). The 2^−ΔCt^ method was used to calculate the mRNA expression levels. ΔCt = Ct_target_ gene − Ct_internal_ control gene (where Ct is the cycle number when the fluorescence signal reaches the set threshold). The amplification parameters were 95 °C for 30 s (95 °C for 5 s, 60 °C for 34 s) for 40 cycles. The analysis was performed with three biological replicates.

#### Western blot

Cells were lysed with RIPA lysis containing protease inhibitor. Cell lysates were collected and the total protein content was estimated by the Bradford method (Bio-Rad). An aliquot of 70 μg of protein extract was loaded in each lane and separated in a 10% SDS-PAGE gel and electroblotted on a PVDF membrane. The membrane was then blocked with 4% BSA in 1× TBS and 0.1% TWEEN®20, washed and probed using antibodies directed against Ezh 2(enhancer of zeste homolog 1), Bmi-1 (B lymphoma mo-MLV insertion region 2), Eed (embryonic ectoderm development), Mll (mixed lineage leukemia), MEL18 (melanoma nuclear protein 18), Rae-28 (polyhomeotic-like protein 1), TOPOIIα (DNA topoisomerase 2-alpha), UHRF1 (ubiquitin-like with PHD and ring finger domains 1), H3K27me3, H3K4me3, and GAPDH (endogenous loading control) overnight at room temperature. Blots were then washed and incubated with (i) 1:2000 dilution of HRP secondary antibody for 2 h at room temperature. The protein bands were developed with chemiluminescent reagents (Millipore). Relative band intensities were determined by using the ImageJ software.

#### Small interfering RNA (siRNA)

Based on significant downregulation of Bmi-1 and Trx in the model group, Bmi-1 and Trx were selected for Small interfering RNA to validate their effect on the target gene UHRF1 and TOPO and aging-related manifestations. Three siRNAs targeting Bmi-1 and Trx were designed and synthesized, respectively. Transfection: Cells were collected and resuspended in HSPCs medium without cytokines; 20 pM of siRNA was added to 50 μl of Opti-MEM serum-free medium; an equivalent amount of irrelevant siRNA was added as a negative control. Mixed the solution above before adding 400 μL of cell suspension (0.5–2 × 10^5^ per well in a 24-well plate) to it. 1.5 μl of Lipofectamin 3000 (Invitrogen) reagent was added with 50 μl of Opti-MEM. After 6 h of incubation at 37 °C/5%CO_2_, the complexes were removed and the cells were incubated with cytokine-free media for up to 48 h after transfection. The mRNA expression levels of Bmi-1, Trx, TOPOIIα, and UHRF1 were detected by real-time fluorescence quantitative PCR. The protein expressions of Bmi-1, Trx, TOPOIIα, and UHRF1 were detected by Western blotting. We also performed SA-β-gal staining and CFU-Mix formation assay to observe aging manifestation.

#### Chromatin immunoprecipitation (ChIP)

The cells were fixed with formamide at a final concentration of 1% to cross-link the H3K4me3 or H3K27me3 with DNA. After the cells were broken by SDS lysis buffer, DNA was sonicated to a size of 250–1000 bp (input DNA). The DNA protein complex was precipitated with specific antibodies (H3K4me3 or H3K27me3), absorbed onto the protein A agar, and decrosslinking. The precipitated DNA fragment was stored at − 20 °C for a long time (this DNA fragment was named ChI Ped DNA). Fluorescent quantitative PCR was used to detect TOPOIIα and UHRF1 levels of ChIPed DNA.

#### Statistical analysis

The experimental data was expressed as a mean and standard deviation. Single-factor analysis of variance and one-way ANOVA were performed using SPSS 18.0. The LSD or Tamhane test was used to compare the differences between the two groups. *p* < 0.05 was considered statistically significant.

## Results

### Purification of HSPCs

We detected HSPC purity by flow cytometry. The purity of Lin^−^Kit^+^ cells was 91.7% (Fig. 1d) (n = 10). It indicated that the sorted HSPCs are highly purified and suitable for subsequent experiments.

### The establishment of old HSPC model

HSPCs isolated from 4-week-old mice were cultured with the modeling medium including Stemspan Stem Cell Media, 10 ng/L IL-3,10 ng/mL IL-6, and 30 ng/mL SCF for 8 days. At day 8, flow cytometry was used to determine the ratio of HSPCs (Lin^−^c-Kit^+^). The results showed that the percentage of Lin^−^c-Kit^+^ cells at day 8 was 86% (Fig. 1d). It suggested HSPCs still have a high proportion at day8 and enough for testing.

### The identification of old HSPC model

To identify the old HSPC model, the following experiments were performed: SA-β-gal staining, cell cycle distribution detection, colony-forming assay, transmission electron microscope (TEM), and RNA-seq bioinformatics analysis. We further identify it by the comparative study on HSPCs isolated from old mouse (18-month-old) and old model HSPCs.

#### The percentage of SA-β-gal stain-positive cells increased

SA-β-gal (senescence-associated-β-galactosidase) is a hallmark of aging that can yield a blue stain in the cytoplasm of aging cells [21, 22]. We found that the percentage of SA-β-gal stain-positive cells increased gradually at days 2, 4, 6, and 8 compared with the young group (Supplementary Fig.S1). Therefore, day 8 was chosen as the optimum time of modeling. The percentage of SA-β-gal stain-positive cells in the model group (day 8) and in the old mouse group were significantly higher than those in the young group (day0) (Fig. 2a, Table 1), P < 0.01, P < 0.05. The percentage of SA-β-gal stain-positive in the model group (day 8) was significantly higher than that in the old mouse group (Table 1), P < 0.01. (Fig. 2a). It indicated that the senescence model group has more senescent HSPCs than the old mouse group.

**Fig. 2:** Model HSPCs showed significant manifestations of aging such as increased β-galactosidase activity, G0/G1 phase arrest, decreased colony-forming capacity, and changes in cell morphology. **a** Photomicrographs of SA-β-gal staining(× 200). The percentage of SA-β-gal stain-positive cells was significantly increased in the model group compared with the young group, n = 10. **b** Flow cytometric analysis of cell cycle distribution. The model HSPCs were arrested in G0/G1 phase compared with the young group, n = 10. **c** Photomicrographs of CFU-Mix. The size and number of CFU-Mix significantly decreased in the model group compared with the young group. **d**. Photomicrographs of TEM. The nuclear membranes of young HSPCs were smooth and flat, chromatin evenly distributed; there were few to no inclusion bodies found in the cytoplasm. But the perinuclear cisternae in the model HSPCs widened, and chromatin edge aggregated. A large number of inclusion bodies appeared in the model HSPCs

**Table 1:** Percentage of SA-β-gal stain-positive HSPCs (% x ± s, n = 10)

Group	Percent
Young group	1.02 ± 0.09
Model group	56.4 ± 5.21**
Old mouse group	7.16 ± 1.14*

*P < 0.05, compared with the young group

**P < 0.01, compared with the young group

#### The percentage of G0/G1 phase cells increased

Previous studies showed that senescent HSPCs were arrested in G0/G1 [7, 18]. In the present study, we found that compared with the young group (41.93 ± 1.95%), the proportion of G0/G1 phase cells in the model group was significantly higher (70.28 ± 2.45%), P < 0.01; the proportion of G0/G1 phase cells in old mouse group (46.59 ± 2.32%) was higher than the young group (41.93 ± 1.95%), P < 0.05, but the degree of increase was lower than the model group (Fig. 2b, Table 2). The proportion of PI (S + G2/M) phase cells was significantly decreased in the model group compared with the young group, P < 0.05 (Fig. 2b, Table 2). These results showed that the senescence model HSPCs were arrested in G0/G1.

**Table 2:** Distribution of cell cycles of HSPCs (x ± s, n = 5)

Group	G0/G1	G2/M	S
Young group	41.93 ± 1.95	12.38 ± 0.20	45.69 ± 2.06
Model group	70.28 ± 2.45*	7.28 ± 0.39*	22.45 ± 1.57*
Old mouse group	46.59 ± 2.32	12.64 ± 0.69	40.77 ± 2.15

*P < 0.05, compared with the young group

#### Colony-forming ability decreased

The capacity to form CFU-mix decreased in HSPC aging process [7, 18]. In our study, young group HSPCs formed erythroid progenitor cells (colony-forming unit-erythroid [CFU-E] and burst-forming unit-erythroid [BFU-E]), granulocyte/macrophage progenitor cells (colony-forming unit-granulocyte, macrophage [CFU-GM]), colony-forming unit-granulocyte (CFU-G) and colony-forming unit-macrophage (CFU-M), multi-potential progenitor cells (colony-forming unit-granulocyte, erythroid, macrophage, megakaryocyte [CFU-GEMM]), B lymphocyte progenitor cells (colony-forming unit-pre-B [CFU-pre-B]), whereas the model group HSPCs only occasionally formed CFU-G (Fig. 2c). Furthermore, p-iodonitro-tetrazolium violet staining of CFU-mix experiment clearly showed that compared with the young group, model HSPCs displayed smaller and fewer colonies (Fig. 2c). The number of CFU-Mix colonies formed by old mouse HSPCs was also reduced than that of the young group, but the degree of reduction was lower than that of the model group. These results revealed that the capacity of colony formation of the model HSPCs decreases significantly.

#### The ultrastructure of HSPCs changed

In order to visualize age-related ultrastructure changes of HSPCs, we explored it by using the TEM method. It showed that the nuclear membrane of young HSPC was smooth and flat; there was homogeneous chromatin distribution and no or few inclusion bodies in the cytoplasm (Fig. 2d). However, the perinuclear cisternae of model HSPCs widened, and the chromatin edge aggregated. A large number of inclusion bodies appeared in the model HSPCs. The presence of inclusion body may be due to the aging of organelles that occurs when biomicromolecules are stored but not digested in the lysozyme, eventually accumulating in the cells to become brown liposarcoma [23, 24]. Old mouse HSPCs show similar but less morphologic changes than senescence model HSPCs (Fig. 2d and Supplementary Fig.S2).

#### Age-related metabolic pathways changed by iTRAQ analysis

In order to study the changes of age-related metabolic pathways, we performed quantitative proteomic analysis based on isobaric tags for relative and absolute quantitation (iTRAQ). The volcano plot (a) and the heatmap (b) was shown in Fig. 3. Gene Ontology (GO) analysis revealed that the aging process increased significantly in model HSPCs compared with the young group (*p* < 0.01; Fig. 3c). GO and Kyoto Encyclopedia of Genes and Genomes (KEGG) analyses consistently showed that the most differentially expressed proteins between the model group and the young group were associated with glycolysis, lysosomal, ribosomal synthesis, and mRNA splicing (*p* < 0.01; Fig. 3c, d, Fig.S3). Glycolysis and lysosomal metabolism were significantly increased whereas ribosomal synthesis, and mRNA splicing were significantly reduced in the model group compared with the young group (Table 3, Fig.S3). Glycolytic metabolism increased in model vs young was consistent with the result of increased glycolysis metabolism in the aging process shown by the previous study [25]. Lysosomal phagocytosis enhanced in model vs young was consistent with the electron microscopy data (Fig. 2d). It may be due to a large number of damaged or aging cells and their metabolites, which are phagocytosed by lysosomes. The data also showed that mRNA splicing-related proteins SR, hnRNP, WBP11, splicing factor 3b, and U2AF1 were significantly decreased in model vs young (Table 3). It indicated that the expression of spliced mRNA was significantly decreased. This conclusion is in line with recent research, which found that SF3B1, U2AF1 mutations led to an imbalance of hematopoietic function [26, 27]. The results manifested that many aging-related metabolic pathways changed in model vs young. In addition, STRING of iTRAQ showed that the common target proteins of PcG family and TrxG family are UHRF1 and TOPO IIα, as shown in Fig. 3e. We validated it later in the paper.

**Fig. 3:** Integrated proteomic and transcriptomic analysis showed significant changes of metabolic processes associated with aging in Model HSPCs. **a** The volcano plot of proteomic, which plots significance versus fold change on the y- and x-axes, respectively, found upregulated and downregulated proteins using t-test. The red color represents the upregulated proteins, and the blue color represents downregulated proteins. **b** The heat map of proteomics showed protein expression levels of the young group and the model group. Color intensity indicates the level of expression, where green signifies low expression and red signifies high expression. **c** Gene Ontology analysis of proteomics, p < 0.05. **d** KEGG analysis of proteomics. Go enrichment (**c**) and KEGG pathway (**d**) analysis showed that glycolysis, lysosomal metabolism, ribosomal synthesis, and mRNA splicing were significantly changed in the model. **e** STRING analysis of proteomics showed that the common target proteins of PcG and TrxG are UHRF1 and TOPOIIa. **f** The scatter plot of transcriptomic: red dots were upregulated, and blue dots were downregulated. **g** Go enrichment analysis of transcriptomics showed genes associated with the stress response, inflammation, lysosomal metabolism, and protein aggregation dominated the upregulated expression profile, while the downregulated profile was marked by genes involved in the preservation of genomic integrity and chromatin remodeling

**Table 3:** Differently expressed genes in the KEGG metabolic pathway (model group/young group)

Accession	Description	Gene name	Fold change ratio
G3UVV4	Hexokinase 1	Hk1	1.2
Q3TRM8	Hexokinase-3	Hk3	1.57
P12382	ATP-dependent 6-phosphofructokinase	Pfkl	0.88
Q9WUA3	ATP-dependent 6-phosphofructokinase platelet type	Pfkp	1.66
P52480	pyruvate kinase	Pkm	1.96
P35486	Pyruvate dehydrogenase E1 component subunit alpha	Pdha1	0.95
O70370	Cathepsin S	Ctss	1.87
O89023	Tripeptidyl-peptidase 1	TPP1	1.71
O35114	Lysosome membrane protein 2	Scarb2	1.82
P11438	Lysosome-associated membrane glycoprotein 1	Lamp 1	1.91
P17047	Lysosome-associated membrane glycoprotein 2	Lamp 2	1.42
P50516	V-type proton ATPase catalytic subunit A	Atp6v1a	1.94
Q9Z204	Heterogeneous nuclear ribonucleoproteins C1/C2	Hnrnpc	0.63
Q923D5	WW domain-binding protein 11	WBP11	0.6
Q921M3	Splicing factor 3b subunit 3	SF3B3	0.81
Q3UJB0	Splicing factor 3b subunit 2	SF3B2	0.62
Q9D883	Splicing factor	U2af1	0.5
Q9Z204	Heterogeneous nuclear ribonucleoproteins C1/C2	Hnrnpc	0.63

#### Transcriptome changes by RNA-seq analysis

To identify transcriptome changes in the model group, we examined the expression of more than 16,800 genes using RNA-seq. This analysis revealed 3717 genes that were upregulated and 3931 genes that were downregulated in the model group vs the young group, which is summarized as a scatter plot (Fig. 3f). As shown in Fig. 3g, the biological process of GO terms associated with the differentially expressed genes was related to aging and lysosomal metabolism, ribosomal synthesis, and mRNA splicing. The result was consistent with our proteomics analysis. When applied to the Up-with-Age gene list, the analysis revealed a large number of enriched categories that have been linked to aging in general, such as NO-mediated signal transduction, the stress response (protein folding) and the inflammatory response, whereas categories enriched for Down-with-Age genes often included those involved in the preservation of genomic integrity, such as chromatin remodeling and DNA repair (Fig. 3f). The result was consistent with Margaret A. Goodell’s study [28]. A small hand-picked list is shown in Table 4 showed the most significant differences in genes in the model group and the young group, consistent with the data of Margaret A. Goodell [28].

**Table 4:** Differently expressed genes selected (model group/young group)

Symbol	Gene name	log_2_FC	Significance
Xab2	XPA-binding protein 2	− 1.02	DNA repair
Sirt3	Sirtuin 3	− 1.04	Chromatin silencing
Sirt	Sirtuin	− 1.57	Chromatin silencing
Rad52	RAD52 homolog	− 1.62	DNA repair
Xrcc3	X-ray repair comp. defective repair in C. hamster cells 3	− 2.32	DNA repair
Eng	Endoglin	− 2.81	TGF-b regulates HSPCs pool size
Blm	Bloom syndrome homolog	− 1.48	DNA repair
Sirt	Sirtuin 2	− 1.57	Chromatin silencing
App	Amyloid beta precursor protein	4	Alzheimer disease, stress response
Selp	Platelet-selectin	2.47	Inflammation, adhesion
Ctsb	Cathepsin B	3.56	APP processing, Alzheimer
Ctsc	Cathepsin C	4.85	Proteolysis, inflammation
Icam1	Intercellular adhesion 1	4.2	Cell-cell adhesion, inflammation
Ctss	Cathepsin S	7.4	Proteolysis, inflammation
Cct6a	Chaperonin subunit 6a (zeta)	1.34	Protein folding
Dnajb6	DnaJ (Hsp40) homolog B6	2.8	Protein folding
Tlr4	Toll-like receptor 4	2.08	Inflammation

### The factor of driving the model HSPC aging

To explore what is the main factor of driving the model HSPC aging we treated the cells with IL3 (10 ng/mL), IL6 (10 ng/mL), SCF (30 ng/mL), media (no IL3, IL6, SCF) or together with each other. We evaluate the aging effects with SA-β-gal staining and the CFU-Mix method. The results showed a significant decrease in colony-forming ability and increase in SA-β-gal activity at IL3 groups compared with the control (medium) group (Fig. 4a, i, j). The cells cultured with IL3 alone or together with IL3 were mainly SA-β-gal-positive and showed a significant decrease in the capacity of colony formation (Fig. 4a–d, i, j). There was no significant change in the colony-forming ability and SA-β-gal activity at the cells cultured with IL6,SCF alone or together with IL6,SCF compared with the control (medium) group (Fig. 4e–j). The previous study reported that the growth of HSC in vitro is strictly dependent on growth factors, in particular, IL3 [29]. López et al. demonstrate that IL-3 contributes to cell survival under oxidative stress, a prominent feature in the aging process [30]. In our study, contrary to these researches that IL3 is a positive factor of HSC growth in vitro or anti-aging of cells, our study showed IL3 can lead HSPC to senescence. However, our study was consistent with Frelin et al.’s study that showed Grb2 was positioned as a key adaptor integrating various cytokines response in cycling HSPC by IL3 signaling pathway [31]. Base on the previous researches and our study, we speculated that IL3 could play a role in activating HSPC senescence.

**Fig. 4:** The factors driving the model HSPC aging. **a**–**h** Photomicrographs of SA-β-gal staining (× 100). The cells cultured with IL3 alone or together with IL3 were mainly SA-β-gal-positive. There was no significant change in the SA-β-gal activity at the IL6,SCF alone group or together with the IL6,SCF group. **i**, **j** Photomicrographs of CFU-Mix. The cells cultured with IL3 alone or together with IL3 showed a significant decrease in colony-forming ability. There was no significant change in the colony-forming ability at the IL6,SCF alone group or together with the IL6,SCF group

### Polycomb/Trithorax system disturbance in HSPC aging process

To understand how cellular memory regulates HSPC aging, we examined the gene expressions of PCG (Ezh2,Bmi-1, Eed, Rae-28, Mel18) and TrxG (Mll and Trx) with real-time PCR and Western blot. Furthermore, we explored the target genes of the PcG/TrxG system and identified two genes, UHRF1/TOPOIIa.

#### The changes of Polycomb/Trithorax genes mRNA expression

The A260/280 ratio of RNA extracted from the HSPCs was 1.8–1.9, indicating high purity of RNA. The mRNA levels of Ezh2, Bmi-1, and Eed, Mll in the model group were significantly lower than that in the young group, *p* < 0.01 (Fig. 5a–d); There are no significant differences in the mRNA levels of Mel18, Rae-28, and Trx (Fig. 5e–g).

**Fig. 5:** Polycomb/Trithorax system disturbance in HSPC aging process. RT-PCR was applied to determine the transcription levels of PcG/TrxG genes (**a**). Western blot was applied to determine the levels of PcG/TrxG proteins and TOP2a,URHF1 (**c**) and H3K4,H3K27 (**b**)

#### The changes of Polycomb/Trithorax genes protein expression

The protein levels of Ezh2, Bmi-1, Eed, and Trx in model HSPCs were significantly lower than young HSPCs (Fig. 5h). Mll was significantly increased in the model group, *p* < 0.05, (Fig. 5h). The protein expressions of Mel18 and Rae-28 were not significantly different in the two groups (Fig. 5h). The data of STRING of iTRAQ might also provide us target genes of Polycomb/Trithorax, UHRF1, and TOPOIIα (Fig. 3e). The protein levels of UHRF1 and TOPOIIα were significantly lower than young HSPCs, *p* < 0.05. (Fig. 5h).

To further explore the possible histone methylation regulation of Polycomb/Trithorax on the target genes, the levels of H3K4me3 (trimethylation of histone H3K4) and H3K27me3 (trimethylation of histone H3K27) were examined. H3K4me3 was known to be involved in gene transcriptional activation which can be catalyzed by TrxG [32, 33], and H3K27me3 is involved in transcriptional repression which can be catalyzed by PcG [34, 35]. The total level of H3K27me3 or H3K4me3 was all significantly downregulated in the model group compared with the young group (*p* < 0.01) (Fig. 5l, j). The grayscale of Western blot showed that the ratio of H3k4me3/H3k27me3 in the young group was 0.6, whereas in the model group, it was 0.36 (Fig. 5i, k). It is not difficult to find the reduction of H3K4me3 plays a leading role in the HSPC aging process. So, whether TOPOIIα /UHRF1, which was significantly downregulated, was regulated by the general reduction of H3K4me3, or by a single factor, the reduction of H3K27me3 or H3K4me3 need to be further elucidated below in our study.

### H3K4me3 of TOPOIIα and UHRF1 promoter decreased in model HSPC

To further validate H3K27me3/H3K4me3 of Polycomb/Trithorax on TOPOIIα/UHRF1, we examined it with CHIP-PCR. The data showed that the level of H3K4me3 in TOPOIIα or UHRF1 promoter was both decreased significantly in the model group (Fig. 6a, b), but there was no significant change in the level of H3K27me3 in TOPOIIα or UHRF1(Fig. 6c, d). Therefore, we speculated that H3K4me3, not H3K27me3, downregulated TOPOIIα/UHRF1.

**Fig. 6:** CHIP-PCR showed H3K4me3 of TOPOIIα and UHRF1 promoter decreased in senescent HSPCs. **a**, **b** The level of H3K4me3 in TOPOIIα/UHRF1 promoter was decreased in aging HSPCs. **c**, **d** There was no significant change in the level of H3K27me3 in TOPOIIα/UHRF1 promoter in aging HSPCs

### Knocking down Bmi-1/Trx downregulated TOPOIIα/UHRF1 expression

To further validate TOPOIIα/UHRF1 was the target gene of PCG/TrxG, we studied the effect of knocking down Bmi-1 in PCG or Trx in TrxG on aging-related manifestations and the gene expressions of TOPOIIα and UHRF1. The results showed that the mRNA level and protein level of Bmi-1 or Trx was both significantly decreased after being transfected with Bmi-1 or Trx-siRNA for 48 h, respectively (p < 0.05) (Fig. 7a–d), indicating that siRNA effectively knocked down Bmi-1 or Trx in HSPCs. The mRNA levels of TOPO2a and UHRF1 were both significantly decreased when Bmi-1 or Trx was knocked down, as shown in Fig. 6e, f, p < 0.05. SA-β-gal-stained cells increased in the Bmi-1 or Trx knocked down group, but there was no significant difference (Fig. 7g, h and Supplementary Table.S1); we speculated that cell aging caused by stress need enough time; colony-forming ability of HSPCs significantly decreased in the Bmi-1 or Trx knocked down group compared with the control group, P < 0.05, (Fig. 5i, j). The results not only demonstrated TOPOIIα and UHRF1 were the target genes of Bmi-1 or Trx in HSPCs, but also indicated Bmi-1 and Trx were important members of PCG/TrxG.

**Fig. 7:** Bmi-1 and Trx were important members of PCG/TrxG protein and knocking down Bmi-1/Trx downregulated TOPOIIα/UHRF1 expression. **a**, **b** HSPCs from 4-week-old mice were transfected with Bmi-1-siRNA and Trx-siRNA at 48 h. Bmi-1 gene expression (**b**, **c**) and Trx gene expression (**a**, **d**) were validated by real-time PCR and WB analysis. mRNA expression of TOPOIIα (**e**) and UHRF1 (**f**) decreased significantly in the Bmi-1 or the Trx knocked down group. SA-β-gal-stained cells increased in the Bmi-1 or the Trx knocked down group, but there was no significant difference (**h**). The colony-forming ability of HSPCs significantly decreased in the Bmi-1 (**j**) or the Trx (**i**) knocked down group compared with the control group

## Discussion

Senescence HSPC model in vitro is an important platform to study HSPC senescence and screen the anti-aging drug for hemopathy. Our study presented a quick and easy method of building senescence HSPC model in vitro with a 4-week mouse. The method had the advantages including shorter time requirements and easy operation.

Our senescence HSPC model showed a significant increase in senescence-related β-gal activity, cell cycle arrest, reduction in colony-forming ability of HSPCs, age-related changes in cell morphology, and age-related metabolic pathway. Furthermore, the model HSPCs showed more obvious aging manifestation compared with the HSPCs of natural aging mouse, so we speculated that this was a model of accelerating HSPC aging in vitro compared with in vivo.

Polycomb group (PcG) and Trithorax group (TrxG) are evolutionarily conserved chromatin-modifying factors identified as histone methyltransferase complexes, which can methylate histone lysine-specific sites of target proteins. The TrxG/PcG system maintains the balance of cellular memory system that prevents the change of stem cells identity by antagonizing each other [36, 37]. In addition, in recent years they were found to have more widely control a plethora of cellular processes. This functional diversity is achieved by their ability to regulate chromatin at multiple levels, ranging from modifying local chromatin structure to orchestrating the three-dimensional organization of the genome. So, understanding the TrxG/PcG system is a fascinating challenge of critical relevance for biology and medicine [38]. PcG proteins assemble in multimeric complexes, PRC1 and PRC2 (Polycomb repressive complexes 1 and 2), and induce transcriptional repression of target genes through chromatin modifications such as H3K27me3 [39, 40]. Conversely, TrxG complex induce transcriptional activation of target genes through chromatin modifications such as H3K4me3 [41]. PRC1 consists of ph 1/Rae-28, Bmi-1, Mel-18, and other proteins in mammals [42]. The primary function of PRC1 is to label mono-ubiquitination of the 119th lysine site of histone H2A, thereby recruit PRC2 complex. PRC2 consists of EeD, Ezh2, Su(z)12, and other proteins induce transcriptional suppression of target genes through chromatin modifications such as H3K27me3 and lysine26 on histone 1 (H1K26 me3) [43]. TrxG is mainly composed of Trx, Ashl, and Mll. The previous study indicated that TrxG and PcG proteins can co-occupy and modify chromatin. TrxG protein-deposited histone modifications such as methylation at H3K4 can block PRC2 action and can, hence, antagonize PcG and counteract gene repression [44]. Our study showed that the levels of PcG (Ezh2, Bmi-1, Eed) and TrxG (Mll, Trx) were significantly changed in aging HSPCs and the changes were accompanied by obvious aging manifestations. It meant that the balance of the TrxG/PcG system in HSPC was affected in the aging process, so HSPC could not remember their own mission to continue differentiating into mature blood cells, hence, caused the aging of HSPC.

Furthermore, Western blot with anti-mouse H3K27me3 McAb and H3K4me3 McAb showed that aging HSPCs had significantly lower levels of H3K27me3 and H3K4me3 compared with young HSPCs. As Petruk S noted in his study, genetically, mutations in trxG and PcG genes can antagonize each other’s function, whereas mutations of genes within each group have synergistic effects [45]. In our study, most of PcG and TrxG proteins were downregulated, thereby we speculated it suppressed the levels of H3K27me3 (by PcG) and H3K4me3 (by TrxG). The data also implied that the regulating effects of PcG/TrxG on the target genes may be mediated by H3K27me3 (by PcG) and H3K4me3 (by TrxG) and need further validation in our study.

About the target genes of PcG/TrxG, Hox genes were reported more frequently. Our ITRAQ STRING data hinted that the common target genes for PcG and TrxG were UHRF1 and TOPOIIα, we did further validation with siRNA and Chip-PCR. UHRF1 (ubiquitin-like with PHD and ring finger domains 1), also known as 90 kDa inverted CCAAT box binding protein (ICBP90) or nuclear phosphoprotein 95 (NP95). UHRF1 controlled the self-renewal versus differentiation of HSCs by epigenetically regulating cell-division modes, suggesting that UHRF1 could affect HSPCs’ fate [46]. Topoisomerase (TOPO) is an enzyme that can cut DNA at a particular point to unravels the DNA twist and relieves the DNA supercoil nature. It plays an essential role during DNA replication. TOPOII (topoisomerase II) catalyze a transient double-strand DNA break, which allows the passage of another DNA duplex through the break before the strands are resealed. There are two isoforms of mammalian TOPOII, TOPOIIα and TOPOIIβ. The study of hematopoietic toxicity suggested that the level of TOPOIIα was decreased in bone marrow mononuclear cells of hematotoxic mice, accompanied by reduced acetylation of histone H4 and histone H3 on TOPOIIα promoter [47]. The previous study also demonstrated that TOPOIIα represents the target enzyme for hematological anticancer drugs, including for leukemias and lymphomas [48]. These studies hinted the important roles of TOPOIIα and UHRF1 in anti-damaged of HSC/HSPC. In the present study, the levels of TOPOIIα and UHRF1 were both significantly downregulated in the aging group. RNA interference on Trx in TrxG or Bmi-1 in PcG downregulated the gene expressions of UHRF1 and TOPOIIα. Meanwhile, it inhibited the colony-forming ability of HSPC. The results not only further indicated TOPOIIα and UHRF1 were the target genes of Bmi-1 or Trx that was important PCG/TrxG proteins in HSPCs, but also hinted the role of TOPOIIα/UHRF1 in anti-damaged of HSPC, it is worthy of verification.

Based on our hypothesis that TOPOIIαand UHRF1 were the target genes of PCG/TrxG in the process of HSPC aging, we need to know if UHRF1 and TOPOIIα were methylated by H3K4me3 or H3K27me3 that was downregulated by TrxG/PCG. CHIP-PCR assay showed that the H3K4me3 levels of TOPOIIα and UHRF1 promoter were lower in aging HSPCs compared with young HSPCs, whereas there was no significant difference in the H3K27me3 levels of TOPOIIα/UHRF1. We speculated that it may contribute to the decreased expression of TOPOIIα/UHRF1 in aging HSPCs because of H3K4me3 positive regulation on target genes [42]. Petruk S noted in his study “no overall synergism or antagonism between the trxG and PcG proteins and, instead, only subsets of trxG proteins act synergistically” [45]. Consistent with his study, our findings demonstrated UHRF1/TOPOIIαwas regulated by H3K4me3 of TrxG.

## Conclusion

In conclusion, our work proposed a quick and easy method of building senescence HSPCs in vitro with 4-week mice which can be used for experimental study of HSPC aging, forecasted that can be used for preliminary screen drugs of hemopathy. On the basis of this model and our preceding work on naturally aged mice, we made the point that TrxG/PcG disequilibrium impaired cellular memory of HSPC, so that HSC/HSPC could not remember their own mission to continue differentiating into mature blood cells, then led finally to cause or aggravate the aging of HSPCs. Our studies further identified UHRF1/TOPOII as target genes of the TrxG/PcG system in the HSPC aging process. TrxG/PcG disequilibrium shown in this paper extended our understanding of the molecular mechanisms underlying HSPC senescence.

## Supplementary Information

**Additional file 1: Fig. S1.** The percentage of SA-β-gal stain-positive cells. The percentage of SA-β-gal stain-positive cells increased gradually at day2, 4, 6, 8.

**Additional file 2: Fig. S2.** The ultrastructure of HSPCs changed. The photomicrographs of TEM showed that nuclear membrane, perinuclear cisternae, chromatin edge, inclusion body in cytoplasm of HSPC changed. Old mouse HSPC showed similar but less morphologic changes than model HSPC.

**Additional file 3: Fig. S3.** Proteomics KEGG pathway analysis of differentially expressed proteins. (a,b), Pyruvate kinase were significantly increased and pyruvate dehydrogenase E1were reduced in the model cells. (c,d), Dkc1, GAR1, Nop10, Nog1 and ribosomal proteins in the ribosome-sized subunits also decreased significantly in the model cells. (e), U2AF1 (U2AF) 1 were significantly decreased in the model cells. (f), Lysosomal related proteins such as Cathepsin, TPP1, lysosomal membrane protein LIMP, lysosomal-associated membrane protein (LAMP), and ATPeV were significantly increased in the model cells.

**Additional file 4: Table S1.** Percentage of SA-β-Gal positive HSPCs (% x ± s, n=3).

## Data Availability

All data needed to evaluate the conclusions in the paper are present in the paper and/or the materials cited herein. Additional data related to this paper may be requested from the authors.

## Abbreviations

HSPC(s): Hematopoietic stem and progenitor cell(s)
MACS: Magnetic cell sorting
CFU: Colony forming unit
TEM: Transmission electron microscope
t-BHP: Tert-butyl hydroperoxide hydroperoxide
PcG: Polycomb group
TrxG: Trithorax group
MNCs: Bone marrow mononuclear cells
Lin: Lineage
IL3: Interleukin 3
IL6: Interleukin 6
SCF: Stem cell factor
SA-β-gal: Senescence-associated beta-galactosidase
RNA-seq: RNA sequencing
iTRAQ: Isobaric tags for relative and absolute quantification
ChIP: Chromatin immunoprecipitation
CFU-E: Colony-forming unit-erythroid
BFU-E: Burst-forming unit-erythroid
CFU-GM: Colony-forming unit-granulocyte, macrophage
CFU-G: Colony-forming unit-granulocyte
CFU-M: Colony-forming unit-macrophage
CFU-GEMM: Colony-forming unit-granulocyte, erythroid, macrophage, megakaryocyte
CFU-pre-B: Colony-forming unit-pre-B
GO: Gene Ontology
KEGG: Kyoto Encyclopedia of Genes and Genomes
Mll: Mixed lineage leukemia
Ezh2: Enhancer of zeste homolog 2
Bmi-1: B cell-specific MLV integration site-1
Trx: Thioredoxin 1
Eed: Embryonic ectoderm development
Mel-18: Pcgf2 polycomb group ring finger 2
Rae-28: Phc1 polyhomeotic-like 1
UHRF1: E3 ubiquitin-protein ligase UHRF1
TOPOIIa: DNA topoisomerase 2-alpha
H3K27me3: Trimethylation of histone H3K27
H3K4me3: Trimethylation of histone H3K4
